The article "Synthesis and Characterization of Banana and Pineapple Reinforced Hybrid Polymer Composite for Reducing Environmental Pollution" was published in 2022. Journal: Bioinorg Chem Appl.

# Synthesis and Characterization of Banana and Pineapple Reinforced Hybrid Polymer Composite for Reducing Environmental Pollution

**DOI:** 10.1155/2022/6344179

**Published:** 2022-05-11

**Authors:** M. Ramesh, D. Jafrey Daniel James, G. Sathish kumar, V. Vijayan, S. Raja Narayanan, Aklilu Teklemariam

**Affiliations:** ^1^Department of Mechanical Engineering, K. Ramakrishnan College of Engineering, Tiruchirappalli, Tamil Nadu, India; ^2^Department of Mechanical Engineering, K. Ramakrishnan College of Technology, Tiruchirappalli, Tamil Nadu, India; ^3^Department of Mechanical Engineering, M. Kumarasamy College of Engineering, Karur, Tamil Nadu, India; ^4^Department of Mechanical Engineering, Faculty of Manufacturing, Institute of Technology, Hawassa University, Hawassa, Ethiopia

## Abstract

Nonbiodegradable polymers constitute major pollution and their usage cannot be ignored due to their properties. Hybrid polymer composite research has increased in recent times due to improved characteristics and biodegradable nature. The effect of different stacking sequences containing pineapple/banana/basalt fiber has been studied in the present work to reduce the usage of synthetic fibers without compromising on properties. Hybrid composites were manufactured using the hand layup method and were assessed for mechanical and morphological characteristics. The results showed that several properties improved by keeping the pineapple layer in the skin layer. The adhesion between the matrix and the fiber played a vital role in determining the properties of the composites manufactured. Morphological studies have concluded that the proper bonding between the matrix and the fiber has enhanced several properties.

## 1. Introduction

Nowadays, synthetic fibers are being replaced by natural fibers all over the world since they are used in many fields. Natural fibers have many advantages, such as low cost, abundant in nature, and being biodegradable [1]. They may be extracted from plants, minerals or animals. Natural fibers derived from plants are commonly used in a number of applications [2]. The characteristics of the natural fiber obtained depend on the place from which the fibers are extracted. The crystalline contents, such as cellulose, and amorphous contents, such as hemicellulose, lignin, and pectin, depend on the conditions under which the plants grow [3]. The amorphous content of natural fibers must be lower, eliminating the need for chemical treatment. Natural fibers are available in a variety of forms such as bi-woven mats or single fiber mats or unidirectional mats. These mats can be combined with different stacking sequences, which are generally referred to as hybridization [4]. Sekran et al. [5] investigated hybrid composites containing *Aloe vera* and sisal fibers. They concluded that hybrid composites resulted in improved mechanical characteristics.

The article "Synthesis and Characterization of Banana and Pineapple Reinforced Hybrid Polymer Composite for Reducing Environmental Pollution" was published in 2022. Journal: Bioinorg Chem Appl.

Sanjay and Yogesha [6] carried out their research work on finding the interlaminar shear and impact properties of E-glass/kenaf/jute fibers with different stacking sequences which were manufactured by the process of vacuum bagging. They concluded that the properties of kenaf/jute fiber were improved when E-glass fiber was kept at the outer ends. Hybrid fibers containing jute, abaca, and glass fibers were manufactured using a hand layup method described by Vijaya Ramnath et al. [7]. As a result, it was concluded that by placing high strength fiber in the middle, the properties improved. Hybrid composites containing *Cyperuspangorei*, jute fibers, and glass fibers at the outer layers were manufactured by the hand layup method [8]. The experimental result showed that, when the jute fiber was kept at the core layer and *Cyperus pangorei* at the intermittent layer, the properties were improved compared to other stacking sequences.

In the previous study, James et al. [9] stacked sisal/bagasse fibers at different stacking sequences and studied their mechanical and morphological properties. Outcomes of the test results revealed that when three layers of sisal were stacked there was an increase in properties. From the vast literature survey, it is also concluded that when there is a proper bonding between the matrix and the fiber there is an increase in several properties. The mechanical properties of the composites containing jute fiber/areca sheath fiber/woven glass fabric which was manufactured by the hand layup method were described by Ganesh et al. [10]. Finally, they concluded that the composites containing areca sheath had improved properties. The mechanical characteristics of sisal and aloe vera composites were studied by Sekaran et al. [5]. Outcomes of the experiment revealed that the hybrid composites have better properties.

From a widespread literature survey, it was found that there were no experimental works on hybrid composites containing basalt, bamboo and pineapple fibers. The present work deals with the manufacturing and characterization of bamboo and pineapple fibers in different stacking sequences, while the basalt fiber was kept in the outer layer in all the composites produced. Mechanical, flammability and morphological characteristics were analyzed for the composites manufactured.

## 2. Materials and Methods

The resin & hardener selected, processing of fibers, manufacturing of composites and characterization techniques are discussed in the following sections.

The article "Synthesis and Characterization of Banana and Pineapple Reinforced Hybrid Polymer Composite for Reducing Environmental Pollution" was published in 2022. Journal: Bioinorg Chem Appl.

### 2.1. Materials

Epoxy resin of grade LY556 was chosen as a binder for the formation of matrix with fibers. The hardener selected was HY951. Both were mixed in the ratio 10 : 1 (Resin: Hardener) for facilitating the polymerization process. At present, a specially designed machine exists for the extraction of banana fibers. It consists of horizontal beams which have a carriage attached to them. It has also a specially designed comb. First, the fibers are placed on a platform which is clamped by jaws. Then it was dried and cleaned at a temperature of 200°C for three hours. Once the process is completed, it is sent to industries for weaving into required patterns. The pineapple fibers are crushed, washed, and brushed with combs to separate the fiber. Finally, the fibers were spun by using chakra. Lastly, it is sent to industries for weaving in a required pattern. Basalt fiber was kept in the outer layer of the composites. In all of the manufactured composites, the basalt fiber is kept at the outer layer. The properties of banana and pineapple fibers are shown in Table 1. All the fibers were obtained from Go green composites, Chennai.

### 2.2. Manufacturing of Composites

Composites containing stacking sequences were manufactured by hand layup process. In the present work, five layers of fibers were with basalt fiber at the outer ends. The other two layers were stacked with banana or pineapple fibers according to the required sequences which are tabulated in Table 2. The different layers of the fibers were manufactured using epoxy resin and hardener with a ratio of 10 : 1. The outer edges were covered with basalt fibers which provide a better load carrying capacity. The stacking sequence carried out is very much similar to Sanjay et al. [11] neglecting the stacking sequence. When the required stacking sequence was completed, a load of 25 kg was applied over the surface and it was cured at room temperature for one day as shown in Figure 1.

### 2.3. Characterization of Manufactured Composites

The tensile strength of the manufactured composites was analyzed according to the ASTM D638-14. The tensile tests were done at a strain rate of 0.5 mm/min using a Universal Testing Machine (Manufacturer: Kalpak, Pune with a capacity of 100 KN). The flexural strength of the manufactured composites was evaluated using the three-point bending test according to ASTM D790-10 at a displacement rate of 2 mm/min. The three-point bending test was carried out with a roller support of size 30 mm. The impact strength of the manufactured composites was estimated according to ASTM D256-10 using a computerized impact testing machine. The specimen size for impact testing is 55 × 55 mm. The hardness of the manufactured composite was measured using Shore D hardness according to ASTM D2250-15. The flammability tests of the composites were carried out according to ASTM D635. The fractured specimen of tensile samples was cut into 10 × 10 mm to study its characteristics. The samples were gold-sputtered to make them conductive. All the tests were carried out thrice, and the average value was noted.

The article "Synthesis and Characterization of Banana and Pineapple Reinforced Hybrid Polymer Composite for Reducing Environmental Pollution" was published in 2022. Journal: Bioinorg Chem Appl.

## 3. Results and Discussions

The composites with designated stacking sequences were manufactured by the hand layup technique. The mechanical and morphological characteristics are discussed in the below sections.

### 3.1. Tensile Strength

The tensile strength of any fiber depends on characteristics such as the strength of the fiber, the orientation in which the fibers are placed and the sequence of the fibers in which they are arranged. Failure during the test depends on how cracks develop on the surface during the test [12].  Figure 2 shows the tensile strength of the manufactured composites. The tensile strength of the C-4 composite was 1.16 times higher than that of the C-2 composite, 1.28 times higher than that of the C-3 composite, and 1.37 times higher than that of the C-1 composite. The tensile strength of the composite C-4 is 282.8 MPa. When the high strength fibers are kept on the layer of the skin, they result in better tensile strength characteristics. Similar kinds of results were reported by Jawaid et al. [12] in the case of oil palm fruit fibers and jute fibers where there is an increase in tensile strength when the high strength jute fibers are kept at the outer layer.

The tensile strength of the fiber depends on the cellulose content of the fiber [13]. When the content of cellulose was higher, the tensile strength increased. In the current study, pineapple fiber has a higher content of cellulose, which is a reason for improving the tensile strength characteristics. This results in a greater degree of polymerization with the matrix and the resistance from tension. A similar increase in tensile strength characteristics was also reported by Islam et al. [14] in the case of kenaf/coir polymer composites in which the higher cellulose content in kenaf resulted in enhanced tensile strength characteristics.

The better bonding between the fiber and matrix also played a vital role in determining the tensile strength characteristics. Jawaid et al. [12] also reported that there is an increase in tensile strength when there is a proper bonding between matrix and fiber. In the case of C-4 composites, there will be a proper bonding between the matrix and fiber as shown in Figure 3(a).

### 3.2. Flexural Strength

The flexural test is usually performed to study the stiffness of the composites. During the flexural testing, the tensile force acts at the bottom, while compression at the top layer and shear at the middle section, which results in higher values when compared to tensile tests. In the case of flexural testing, most of the stress is carried by the outer layer. The proper bonding between fiber and matrix also results in increase in flexural strength [15]. The flexural strength of the manufactured composite is shown in Figure 4. The flexural strength of the C-4 composite is more followed by C-3, C-2, and C-1 composites. The raise in flexural properties of the C-4 composite is due to the good adhesion between the fibers and the matrix. During the flexural testing, the outer layer undergoes tensile stress while the inner layer undergoes compressive stress. The presence of high strength fiber at the skin layer results in more flexural strength values. The observed results also get matched with the results suggested by Nampoothiri et al. [16]. The presence of higher moisture content in banana fiber resulted in less flexural strength values in the case of C-1 composites. The presence of moisture content makes the bonding between the fibers a weaker one and makes delamination easier which results in poor flexural strength values as shown in Figure 3(b). Jawaid et al. [17] also concluded that placing high strength fiber at the skin layer increases the flexural strength considerably.

The article "Synthesis and Characterization of Banana and Pineapple Reinforced Hybrid Polymer Composite for Reducing Environmental Pollution" was published in 2022. Journal: Bioinorg Chem Appl.

### 3.3. Impact Strength

The impact nature of any composite depends on the energy absorbed during the fracture. The Izod impact test was used to measure energy-absorbing characteristics. The energy absorbed by a composite depends on factors such as chemical composition of the fiber, the interface between the matrix and the fiber, the sequence of stacking, and the conditions for testing [18]. Pure fiber has better energy-absorbing properties in all directions as the stacking sequence is made up of the same fiber [19]. The energy absorbed by the manufactured composite is shown in Figure 5. Figure 5 shows that the C-2 composite has higher energy-absorbing characteristics before it breaks down. The results obtained are very similar to those reported by Devi et al. [20] where pure pineapple fiber has improved energy-absorbing characteristics. In the case of C-1 composite, the energy absorbed is much less which makes it necessary to stack the fiber. Jothibasu et al. [18] also suggested that the fibers with less energy-absorbing capacity could be improved by hybridizing them. When banana fiber is hybridized with pineapple fiber, there is an improvement in energy-absorbing properties. In the current study, the composite C-4 manufactured is suitable for energy-absorbing properties due to the increased amount of pineapple fibers in the composite. From the previous literature survey, it can be concluded that the impact is also dependent on the manufacturing process and from where the fiber is extracted.

The article "Synthesis and Characterization of Banana and Pineapple Reinforced Hybrid Polymer Composite for Reducing Environmental Pollution" was published in 2022. Journal: Bioinorg Chem Appl.

### 3.4. Shore D Hardness

The term hardness is defined as surface indentation resistance.  Figure 6 shows the Shore D hardness of the manufactured composites. In the current study, the C-1 composite has a higher level of Shore D hardness. The Shore D hardness of the C-1 composite is more due to the presence of stiffer banana fiber at the core and outer layers which prevents the indentation resistance. Similar results have also been reported by Bharath et al. [21].

### 3.5. Flammability Tests

The flammability of the composites depends on the chemical nature of the fiber and its properties. Fiber decomposition occurs when exposed to heat. The flammability test values for the manufactured composites are shown in Figure 7. Both the selected fibers have a meager amount of difference in the cellulose content.  Figure 6 shows that C-2 composites are more flammable resistant. The presence of more moisture content is the primary reason for the increase in flammability properties. The order of flammability characteristics are C-2, C-4, C-3 and C-1 composites. Among the manufactured composites, the composite C-1 was more resistant to flammability due to the presence of more amount of moisture content in the composite [22, 23].

### 3.6. Morphological Characteristics

Figure 3(a) shows the SEM image of the C-4 composite. There is a better bonding between the matrix and the fiber which improved the tensile characteristics. This property has resulted C-4 composite as the best one among the other manufactured composites. Figure 3(b) shows the SEM image of the C-1 composite. A similar kind of increase in strength due to the better bonding between matrix and fiber was also reported by Ramnath et al. [7]. The presence of less amorphous content in the case of C-4 composites resulted in better bonding characteristics. The banana fiber showed more pull out and debonding when compared with pineapple fibers. Due to this debonding and pull out of fibers there was a decrease in several properties. The decrease in properties is also due to more amount of amorphous content which reduced the bonding nature of fiber also leading to a decrease in properties. Due to this debonding, the presence of cracks and voids can be seen on the surface. Vijay and Singaravelu [8] also reported that there was a decrease in properties when there is poor bonding between matrix and fiber. Thus, the output of morphological characteristics gets matched with the experimental results.

The article "Synthesis and Characterization of Banana and Pineapple Reinforced Hybrid Polymer Composite for Reducing Environmental Pollution" was published in 2022. Journal: Bioinorg Chem Appl.

## 4. Conclusion

The hybrid composite containing basalt/pineapple/banana was manufactured by hand layup techniques. The manufactured composites were analyzed for mechanical and morphological characteristics.

- When pineapple fiber was placed in the skin layer and banana fiber in the core layer there was an increase in tensile and flexural characteristics which was due to the presence of high strength at the skin layer. The decrease in tensile and flexural characteristics was due to the improper adhesion between the matrix and fiber.
- The impact strength was more when the pineapple fiber was kept al three layers. When the banana fiber was kept at the three layers, there was a decrease in impact strength values which makes the hybridization essential in the case of banana fiber.
- The values of Shore D hardness were more when banana fiber was reinforced at three layers. The presence of stiffer banana fiber resisted the indentation.
- The flammability characteristics were less when three layers of banana fibers were hybridized. The presence of more amount of moisture content resisted the increase in flammability characteristics.
- SEM studies revealed that when there was a proper bonding between the matrix and fiber, there was an enhancement in properties. When there was fiber debonding and pull out of fibers, there was a decrease in properties which is evident from acquired experimental results.
- This work can be extended by chemically treating fibers through different treatments and stacking them in different sequences and studying their final properties.

## Figures and Tables

**Figure 1:** Process sequence of composite flow chart.

**Figure 2:** Tensile strength of manufactured composites at stated proportions.

**Figure 3:** (a) SEM image of C-4 composite. (b) SEM image of C-1 composite.

**Figure 4:** Flexural strength of manufactured composites at stated proportions.

**Figure 5:** Impact strength of manufactured composites at stated proportions.

**Figure 6:** Shore D hardness of manufactured composites at stated proportions.

**Figure 7:** Flammability of manufactured composites at stated proportions.

**Table 1:** Properties of banana and pineapple fibers.

Sl. No.	Properties		Banana fibers	Pineapple fibers
1	Chemical composition (wt. %)	Cellulose	69.5	74.24
		Hemicellulose	15	12.6
		Lignin	5.45	7.14
		Moisture	13	10
2	Tensile strength (MPa)	529	680

**Table 2:** Composites stacking sequence with designation.

Sl. No	Designation	Stacking sequence
1	C-1	Basalt-banana-banana-banana-basalt
2	C-2	Basalt-pineapple-pineapple-pineapple-basalt
3	C-3	Basalt-banana-pineapple-banana-basalt
4	C-4	Basalt-pineapple-banana-pineapple-basalt

The article "Synthesis and Characterization of Banana and Pineapple Reinforced Hybrid Polymer Composite for Reducing Environmental Pollution" was published in 2022. Journal: Bioinorg Chem Appl.

## Data Availability

The data used to support the findings of this study are included in the article. Should further data or information be required, these are available from the corresponding author upon request.
